The article "Surface modified composite nanofibers for the removal of indigo carmine dye from polluted water" was retracted in 2025. Reasons: duplicated images; unreliable data; unreliable results or conclusions.

# Surface modified composite nanofibers for the removal of indigo carmine dye from polluted water

**DOI:** 10.1039/c8ra02463d

**Published:** 2018-07-10

**Authors:** M. G. Yazdi, M. Ivanic, Alaa Mohamed, A. Uheida

**Affiliations:** Department of Applied Physics, KTH Royal Institute of Technology Stockholm Sweden alakha@kth.se salam@kth.se +201069676710 +46-8-7909132; Division for Marine and Environmental Research, Ruder Boskovic Institute Zagreb Croatia; Egypt Nanotechnology Centre, EGNC, Cairo University 6th October City 12588 Egypt; Membrane Technology Department, Institute of Functional Interfaces (IFG), Karlsruhe Institute of Technology (KIT) 76344 Germany; Production Engineering and Printing Technology Department, Akhbar El Yom Academy 12655 Giza Egypt

## Abstract

Surface coated magnetite nanoparticles (Fe_3_O_4_ NPs) with 3-mercaptopropionic acid were immobilized on amidoximated polyacrilonitrile (APAN) nanofibers using electrospinning followed by crosslinking. The prepared composite nanofibers were characterized with Scanning Electron Microscopy (SEM), and Fourier Transform Infrared analysis (FTIR). The composite nanofiber was evaluated for the removal of indigo carmine dye from aqueous solutions. The effects of contact time, initial dye concentration, solution pH and adsorption equilibrium isotherms were studied. The adsorption of indigo carmine was found to be greatly affected by solution pH. The maximum loading capacity was determined to be 154.5 mg g^−1^ at pH = 5. The experimental kinetic data were fitted well using a pseudo-first order model. The adsorption isotherm studies showed that the adsorption of indigo carmine fits well with the Langmuir model. The reuse of the composite nanofiber was also investigated in which more than 90% of indigo carmine was recovered in 5 min. The results of stability studies showed that the adsorption efficiency can remain almost constant (90%) after five consecutive adsorption/desorption cycles.

## Abstract 2

Surface coated magnetite nanoparticles (Fe_3_O_4_ NPs) with 3-mercaptopropionic acid were immobilized on amidoximated polyacrilonitrile (APAN) nanofibers using electrospinning followed by crosslinking.

## Introduction

The textile industry is one of the major sources of wastewater containing organic dyes. Indigo carmine (IC), also known as 5,5′-indigodisulfonic acid sodium salt, is one of the important organic dyes because its extensive use in textile and other industries such as paper, plastic, leather, food, cosmetics, and printing. These organic dyes are common water pollutants and may cause damage to health and ecosystems due to their mutagenic and carcinogenic effects.^1^ Therefore, there is an urgent need for the removal of these organic dyes from waste effluents. Several techniques have been investigated for the treatment of water streams containing organic dyes, including decolouration, chemical coagulation and precipitation, biodegradation, membrane filtration and active sludge, and adsorption.^2–6^ Among these techniques, adsorption is one of the most efficient processes, and is widely used since the other techniques require a large quantity of chemicals and/or high energy, and are expensive.^7^

The article "Surface modified composite nanofibers for the removal of indigo carmine dye from polluted water" was retracted in 2025. Reasons: duplicated images; unreliable data; unreliable results or conclusions.

There are several materials that have been investigated for the removal of indigo carmine from solutions, including activated carbon,^8^ natural materials^9–12^ and synthetic resins.^13^ Application of some of these materials is limited due to high cost, difficulty of disposal and reuse. In addition, separation of these adsorbents from the aqueous solutions is still problematic.

Recently, composite nanofibers attracted great attention in wastewater treatment applications due to their large surface area to weight ratio, high flexibility, high porosity, and ease of surface functionalization.^14,15^ Previously, we have investigated the use of composite nanofibers for the adsorption of heavy metals^16,17^ and photocatalytic degradation of organic pollutants under UV and visible light irradiation.^18,19^ Furthermore, in our earlier work we have also demonstrated that Fe_3_O_4_ nanoparticles have high potential to be used as adsorbents, either in the form of pristine nanoparticles or after modifying the surface with organic reagents.^20–22^ However, separation of the nanoparticles (adsorbent) from the treated solution limits the process development. One of the plausible strategies is to immobilize the nanoparticles on a flexible substrate such as nanofibers in order to eliminate the nanoparticles separation and their loss to the environment. This will also allow the reuse of the adsorbent material several times on continuous flow system. In this study, composite nanofibers consisting of amidoximated polyacrylonitrile nanofibers (APAN) and surface coated Fe_3_O_4_ nanoparticles with 3-mercaptopropionic acid (3-MPA) were used for the removal of indigo carmine from aqueous solutions. The surface modified Fe_3_O_4_ nanoparticles were chemically cross-linked to the electrospun APAN nanofibers in order to increase the density of active adsorption binding sites and thus improve the adsorption efficiency of the organic dye.

## Materials and methods

### Reagents and chemicals

Polyacrylonitrile (PAN) (molecular weight, MW = 10 121), hydroxylamine hydrochloride (NH_2_OH·HCl), sodium carbonate (Na_2_CO_3_), were purchased from Sigma Aldrich. *N*-Hydroxysuccinimide (98%-NHS), 1-ethyl-3-(3-dimethylaminopropyl)carbodiimide (EDC), iron(ii) chloride tetrahydrate (FeCl_2_·4H_2_O), iron(iii) chloride hexahydrate (FeCl_3_·6H_2_O), diethylene glycol (DEG), dimethylformamide (DMF), sodium hydroxide (NaOH), nitric acid (HNO_3_), ethanol and 3-mercaptopropionic acid (3-MPA) was purchased from Sigma Aldrich., and deionized water (DI) with resistivity of 15 MΩ cm using Mili-Q water was used in all experiments. Indigo carmine (C_16_H_8_N_2_Na_2_O_8_S_2_) was purchased from Sigma Aldrich and used without further purification. The color index numbers (CI) of indigo carmine dye is 73 015. The chemical structure of indigo carmine is shown in Fig. 1.

The article "Surface modified composite nanofibers for the removal of indigo carmine dye from polluted water" was retracted in 2025. Reasons: duplicated images; unreliable data; unreliable results or conclusions.

**Fig. 1:** Chemical structure of indigo carmine dye.

### Preparation of the adsorbent

PAN/DMF solution, with concentration of 10 wt% was prepared by stirring at room temperature to obtain a homogenous solution. The spinning solution was kept in a vertical syringe with stainless steel needle having an orifice of 0.8 mm. Electrospinning was carried out in an insulated box at room temperature at a high voltage of +10 kV. The flow rate of the solution was maintained at 0.5 mL h^−1^. The excess solvent was removed by drying the electrospun PAN nanofibers in vacuum.^23^

APAN nanofibers were prepared as detailed elsewhere.^24^ The nanofibers were placed into 100 mL solution containing a mixture of 8 g NH_2_OH·HCl, and 6 g of Na_2_CO_3_. The reaction was carried out at 30 °C for 24 h. The nanofibers were then washed three times with distilled water in order to remove the remaining salts and were air dried. The surface functionalization of Fe_3_O_4_ nanoparticles with thiol group was carried out using ligand exchange method.^25^ Subsequently, 0.5 mmol of FeCl_2_·4H_2_O, 1 mmol of FeCl_3_·6H_2_O and 20 g of diethylene glycol (DEG) were added to a three-necked flask with nitrogen bubbling through the solution and flask environment. A mixture of 4 mmol of NaOH and 10 g of DEG was then added to the flask. The mixture was heated to 220 °C and kept under constant stirring for 2 h. 1 mmol of capping ligand (3-MPA) was dissolved in a mixture of 400 μL DI water and 5 g DEG. After two hours, this mixture was injected into the flask and then the system was cooled to room temperature while constantly stirring. The product was then washed 5 times with ethanol followed by centrifugation at 8000 rpm for 10 min in order to remove the excess of DEG and other unreacted chemicals. Finally, the nanoparticles were re-dispersed in DI water.

The surface of the functionalized Fe_3_O_4_–MPA nanoparticles were then activated using (1-3-dimethylaminopropyl)-3-ethylcarbodiimide hydrochloride (EDC)/*N*-hydroxysuccinimide (NHS) to be further coupled to the surface of APAN nanofibers containing the primary amine functional sites. An aqueous dispersion (2 mL) of as-synthesized 3-MPA capped Fe_3_O_4_ nanoparticles were added to 95.8 mg of EDC and 57.5 mg of NHS dissolved in 100 mL sulphate buffer solution. The solution was shaken for 30 min at room temperature. The surface activated Fe_3_O_4_–MPA nanoparticles were then added to APAN nanofibers and kept shaking for 3 h to fulfill the crosslinking reactions. The final composite nanofibers were washed with DI water for 3 times to remove the uncoupled nanoparticles and reaction by-products. The composite nanofibers were dried in air at room temperature. A schematic representation of the aforementioned process based on the fabricated composite nanofibers is briefly sketched (Fig. 2).

The article "Surface modified composite nanofibers for the removal of indigo carmine dye from polluted water" was retracted in 2025. Reasons: duplicated images; unreliable data; unreliable results or conclusions.

**Fig. 2:** Schematic representation of the fabrication process of APAN/Fe_3_O_4_–MPA composites nanofiber.

### Characterization

Morphology of the nanofiber composites was observed using scanning electron microscopy (SEM, Zeiss Ultra 55) equipped with energy-dispersive X-ray (EDX) detector. Fourier transform infrared spectroscopy (FT-IR, Nicolet iS10) was used to confirm the presence of thiol groups on the surface of the nanoparticles as well as the covalent attachment of nanoparticles onto the surface of the nanofibers. The concentration of IC in the solution was measured using UV-Vis/NIR spectrophotometer (model LAMBDA 750, Perkin Elmer) at the maximum absorption wavelength (*λ*_max_) of 611 nm.

### Adsorption/desorption experiments

Adsorption and desorption of IC dye from aqueous solutions were performed using batch operation modes at room temperature. The effect of contact time, solution pH, and initial dye concentration on adsorption were investigated. To study the effect of contact time on adsorption, a solution of IC with initial concentration of 20 mg L^−1^ was continuously mixed with the composite nanofibers and samples were withdrawn in fixed intervals of time for analysis.

Adsorption kinetics was conducted using the batch method. The experiments were carried out in 250 mL glass flask containing a fixed amount of adsorbent of 10 mg with 100 mL dye solution at initial concentration of 20 mg L^−1^. The nanofibers mat was placed on an acrylic support with size of 6 cm × 6 cm to facilitate the separation of the nanofibers mat from the dye solution. The initial pH of the solution was adjusted with 0.1 mol L^−1^ HNO_3_ or 0.1 mol L^−1^ NaOH solutions by using a pH meter. The flask was agitated using orbital shaker (model KS 260, IKA). Liquid samples were taken at regular time intervals and the concentration of dye in the solution was analyzed using UV-Vis/NIR spectrophotometer. The wavelength used for the analyses was 611 nm.

The article "Surface modified composite nanofibers for the removal of indigo carmine dye from polluted water" was retracted in 2025. Reasons: duplicated images; unreliable data; unreliable results or conclusions.

The IC adsorption isotherms for the fabricated composite nanofibers were measured by varying the initial dye concentrations and keeping the other conditions constant. Thus the composites nanofibers were in contact with 10 mL of aqueous solutions with different initial dye concentration (5–100 mg L^−1^) at room temperature. The solutions were mixed with the composite nanofibers for 2 hours at pH = 5. After adsorption, the amount of residual dye in the solution was measured through UV-Vis spectrophotometer. The equilibrium adsorption capacity of APAN/Fe_3_O_4_–MPA was calculated according to the following equation;

1 *q*_e_ = (*C*_i_ − *C*_e_)*V*/*m*

Where *q*_e_ is the amount adsorbed (mg dye/g adsorbent) at equilibrium, *C*_i_ is the initial dye concentration (mg L^−1^), *C*_e_ is the final dye concentration (mg L^−1^), *V* is the solution volume (L) and *m* is the mass of adsorbent used (g).

Desorption of IC was carried out by mixing the loaded composite nanofibers with 4 mmol L^−1^ NaOH aqueous solution in which the final eluting solution was at pH = 10. Samples of IC were withdrawn at fixed intervals of time for analysis. The desorption efficiency of IC from the nanofibers composites was calculated using the following expression;

2 %Desorption = (*C*_des_/*C*_ads_) × 100

where *C*_des_ is the amount of IC released into the aqueous solution (mg L^−1^), and *C*_ads_ is the amount of IC adsorbed onto the composite nanofibers (mg L^−1^).

## Results and discussion

### Adsorbent characterization

SEM micrographs of APAN/Fe_3_O_4_–MPA are shown in Fig. 3. The diameter of the as-prepared electrospun APAN nanofibers (Fig. 3a and b) was determined to be 135 ± 12 nm. Fig. 3c shows the SEM image of the final composite nanofibers. It can be clearly seen that Fe_3_O_4_ nanoparticles are attached to the surface of APAN nanofibers. The surface of APAN/Fe_3_O_4_–MPA composite nanofibers did not show any serious cracks or degradation.

**Fig. 3:** SEM images of (a) APAN nanofibers (b) APAN nanofibers size distribution, (c) APAN/Fe_3_O_4_–MPA composites nanofiber.

FTIR spectra of APAN nanofibers and APAN/Fe_3_O_4_–MPA composites nanofiber were obtained and the results are presented in Fig. 4. The spectrum for APAN exhibited characteristic peaks of nitrile (2242 cm^−1^), carbonyl (1660 cm^−1^), C–H stretching (2941 cm^−1^) and CH_2_ bending (2870 cm^−1^). It can be observed the characteristic peaks of 969 cm^−1^ (assigned to N–O), and the bending vibrations of the amine group NH or NH_2_ (1667 cm^−1^) confirms the conversion of the nitrile group to amidoxime. The shoulder at 1600 cm^−1^ is assigned to N–H bond, which is due to presence of amine groups after functionalization.^26^ Peak at 1653 cm^−1^ is also attributed to both N–H and N–O groups present at both APAN and APAN/Fe_3_O_4_–MPA.^27^ However, the reason for the shift and higher intensity of the peak for APAN/Fe_3_O_4_–MPA is due to the presence of amide groups with strong absorption about 1640 cm^−1^, produced by chemical reaction between carboxyl groups of nanoparticles and primary amine of the nanofibers. The overlapping between broad band of N–O and N–H with strong band for amide has been observed as a single band at 1649 cm^−1^.^28^ The band at 915 cm^−1^ assigned to N–O, demonstrate that the surface functionalization of the nanofibers has been completed. The presence of CH_2_ and C=O peaks, which further prove the presence and successful bonding of iron oxide nanoparticles to the surface of the nanofibers.^29^ The C–S spectra band, which is between 600 to 700 cm^−1^ overlaps with the iron oxide vibrational band and it would be hard to distinguish.^30,31^ The peak at 1700 cm^−1^, which is assigned for stretching of C=O carboxylic group has disappeared from the spectra and instead the peak at 1650 cm^−1^ has become sharper with high intensity. This suggest that the binding of 3-MPA to Fe_3_O_4_ nanoparticles occurs by formation of surface bonds through the COOH group rather than through the SH group. Similar observations were reported for ZnO coated with 3-mercaptopropionic acid^32^ and iron oxide nanoparticles coated with mercaptosuccinic acid.^33^

The article "Surface modified composite nanofibers for the removal of indigo carmine dye from polluted water" was retracted in 2025. Reasons: duplicated images; unreliable data; unreliable results or conclusions.

**Fig. 4:** FTIR spectra of (a) PAN nanofibers, (b) APAN nanofibers, and (c) APAN/Fe_3_O_4_–MPA.

### Adsorption kinetic

The contact time between the adsorbate and adsorbent plays an important role for the removal of pollutants from contaminated waters. The time needed to attain equilibrium was determined by studying the effect of the contact time on the adsorption equilibrium of IC onto APAN/Fe_3_O_4_–MPA. The effect of the contact time was studied under pH = 5 and IC concentration of 20 mg L^−1^ at room temperature (23 ± 1 °C). The results obtained (Fig. 5) showed that the adsorption of IC molecules on the surface of APAN/Fe_3_O_4_–MPA was initially fast enough to remove about 60% of IC in 5 min. Then a gradual decrease in the adsorption rate leading to pseudo equilibrium which was achieved in less than 25 min of contact time with more than 95% of IC adsorbed. Therefore, the rate of adsorption of IC was fast in the initial stage of the process, but gradually reaches a plateau indicating saturation in which equilibrium is reached in 25 min.

**Fig. 5:** Contact time as a function of the adsorption capacity for IC onto APAN/Fe_3_O_4_–MPA. The solid and dashed lines represent non-linear pseudo-first order model and pseudo-second order model fitting to the experimental data. Experimental conditions: dye initial concentration = 20 mg L^−1^, adsorbent amount = 10 mg, pH = 5. The relative standard deviations of all measurements were less than 5%.

The article "Surface modified composite nanofibers for the removal of indigo carmine dye from polluted water" was retracted in 2025. Reasons: duplicated images; unreliable data; unreliable results or conclusions.

The rapid adsorption rate may be attributed to the presence of large number of available active binding sites (–SH) on Fe_3_O_4_ nanoparticles surface, large surface area, and/or higher intrinsic reactivity of the surface sites, which leads to bind more dyes molecules and consequently decrease in the concentration of adsorbate in the solution. As the equilibrium is attained the binding active sites on the surface of Fe_3_O_4_–MPA nanoparticles reach saturation. Various sorbents such as activated carbon,^34,35^ charcoal from coffee beans and rice bran,^36,37^ chitosan,^38^ silica gel,^39^ and activated sewage sludge,^40^ adsorbed IC from aqueous solutions within 2 h to 7 days. In this study, the short equilibrium time suggests that surface modified APAN/Fe_3_O_4_–MPA have high potential to adsorb toxic dyes from aqueous solutions, which would be helpful in lowering the capital and operational costs for industrial applications.

To pinpoint the rate-controlling mechanism of the adsorption of IC onto APAN/Fe_3_O_4_–MPA, the experimental data was fitted using the non-linear regression of pseudo-first order, pseudo-second order, general-order kinetic, and the Avrami kinetic models. In this study, non-linear method was used to determine the kinetic parameters by minimizing the respective coefficient of determination between experimental data and predicted values. The non-linear expressions of pseudo first-order and pseudo second-order kinetic models are given in eqn (4) and (5), respectively;^41^

3 *q*_*t*_ = *q*_e,cal_(1 − exp^−*k*_1_*t*^)

4

The initial adsorption rate can be expressed by;

5 *h* = *k*_2_*q*_e,cal_^2^

The general order kinetic, and the Avrami models can be described by the following equations, respectively;^42^6

7 *q*_*t*_ = *q*_e,cal_{1−exp[−(*k*_AV_*t*)]^*n*_AV_^}

where *k*_1_ (min^−1^) is the pseudo-first order rate constant of adsorption, and *k*_2_ (min^−1^) is the pseudo-second order rate constant of adsorption, *t* is the contact time (min), *k*_N_ is the general order rate constant [min^−1^ (g mg^−1^)^n−1^], *n* is the order of adsorption; *k*_AV_ is the Avrami kinetic constant (min^−1^); and *n*_AV_ is the fractional adsorption order related to the adsorption mechanism, while *q*_e,cal_ and *q*_*t*_ (mg g^−1^) are the calculated (theoretical) adsorption capacity at equilibrium, and adsorption capacity at time *t*; respectively.

The article "Surface modified composite nanofibers for the removal of indigo carmine dye from polluted water" was retracted in 2025. Reasons: duplicated images; unreliable data; unreliable results or conclusions.

In this study, the coefficient of determination (*R*^2^), adjusted coefficient of determination (*R*_adj_^2^), and the standard deviation (SD) was used to test the best-fitting of the kinetic model to the experimental data:8910where *q*_i_,_cal_ represents the individual theoretical *q* value predicted by the model; *q*_i,exp_ represents the individual experimental *q* value; *q̄*_exp_ is the average of experimental *q* values; *n* represents the number of experiments; and *p* represents the number of parameters in the model^45^

Fig. 5 shows the adsorption experimental data and the predicted pseudo first-order, pseudo second-order, general-order, and the Avrami kinetic models. The obtained values of the kinetic parameters are given in Table 1; high adjusted coefficients of determination and low standard deviations indicate good agreement between the experimental and theoretical results.^45^ The higher *R*_adj_^2^ and lower SD values for pseudo first-order kinetics suggest this model can be used to represent the adsorption kinetic of IC onto APAN/Fe_3_O_4_–MPA. It was also observed that the pseudo first-order kinetics predicts the *q*_e,cal_ value more accurately, suggesting the applicability of the model in representing the IC adsorption by APAN/Fe_3_O_4_–MPA at equilibrium conditions.

**Table 1:** Kinetic parameters for the sorption of IC onto APAN/Fe_3_O_4_-MPA obtained using the nonlinear method

**Experimental**
Temperature (K) = 296
**Amount adsorbed at equilibrium**, *q*_e,exp_ (mg g^−1^) = 154.5
Initial IC concentration, (mg L^−1^) = 20
Mass of adsorbent, (mg) = 10
pH = 5

**Model fitting**
**Pseudo-first order model**
Pseudo-first order rate constant, *k*_1_ (min^−1^) = 0.117
Amount adsorbed at equilibrium, *q*_e,cal_ (mg g^−1^) = 153.54
Adjusted determination coefficient, *R*_adj_^2^ = 0.9946
Standard deviation, SD (mg g^−1^) = 0.86

**Pseudo-second order model**
Pseudo-second order rate constant, *k*_2_ (g mg^−1^ min^−1^) = 1.3 × 10^−3^
Amount adsorbed at equilibrium, *q*_e,cal_ (mg g^−1^) = 159.32
Initial sorption rate, *h* (mg g^−1^ min^−1^) = 33
Adjusted determination coefficient, *R*_adj_^2^ = 0.9692
Standard deviation, SD (mg g^−1^) = 4.35

**General order model**
General order constant rate, *k*_N_ [min^−1^ (g mg^−1^)^n−1^] = 0.9186
Amount adsorbed at the equilibrium, *q*_e,cal_ (mg g^−1^) = 164.64
Order of kinetic adsorption, *n* = 1.02
Adjusted determination coefficient, *R*_adj_^2^ = 0.9646
Standard deviation, SD (mg g^−1^) = 8.36

**Avrami model**
Avrami kinetic constant, *k*_AV_ (min^−1^) = 0.1699
Amount adsorbed at the equilibrium, *q*_e,cal_ (mg g^−1^) = 152.77
Fractional adsorption order, *n* = 0.696
Adjusted determination coefficient, *R*_adj_^2^ = 0.9929
Standard deviation, SD (mg g^−1^) = 2.04

The article "Surface modified composite nanofibers for the removal of indigo carmine dye from polluted water" was retracted in 2025. Reasons: duplicated images; unreliable data; unreliable results or conclusions.

### Adsorption isotherms

The equilibrium adsorption capacity of APAN/Fe_3_O_4_–MPA was determined by investigating the effect of initial IC concentration in solution on the adsorbed amount of IC dye per weight of adsorbent at room temperature and pH = 5. The results obtained are illustrated in Fig. 6. The experimental results were fitted using Langmuir, Freundlich, and Toth models. To explain the experimental data non-linear regression analysis was used to estimate isotherm parameters and establish the best-fitting of the isotherm model to the experimental data. Similar to the fitting of the kinetic data (eqn (8)–(10)), the coefficient of determination (*R*^2^), adjusted coefficient of determination (*R*_adj_^2^), and the standard deviation (SD) was used to obtain the best model of isotherm explaining the adsorption experimental data.

**Fig. 6:** Equilibrium isotherm models for the adsorption of IC onto APAN/Fe_3_O_4_–MPA. The solid and dashed lines are Langmuir, Freundlich, and Toth models fit of the experimental data using non-linear method. Experimental conditions: adsorbent amount = 10 mg, contact time = 60 min, pH = 5, temperature = 23 °C ± 1. The relative standard deviations of all measurements were less than 6%.

The Langmuir model assumes the adsorption of IC occurs as a monolayer on a homogeneous surface and is expressed as;11where *K*_L_ (L mg^−1^) is the Langmuir equilibrium constant which is related to the affinity of binding sites with the adsorbate and *q*_m_ (mg g^−1^) is the monolayer capacity referred to the amount of IC required to occupy all the available sites per unit mass of sample. Langmuir isotherm determines whether the adsorption is favorable or unfavorable.

The values of Langmuir parameters obtained from the treatment of the experimental data as well as of the adjusted coefficient of determination (*R*_adj_^2^) and the standard deviation (SD) are listed in Table 2. The high value of *R*_adj_^2^ (0.9820) and low value of SD (3.89) indicated that the adsorption data followed Langmuir isotherm model and the adsorption of IC preferably follows monolayer and homogeneous adsorption process. The calculated maximum adsorption capacity for IC (152.35 mg g^−1^) obtained in this work in comparison with other reported adsorbents was listed in Table 3.

**Table 2:** Isotherm parameters obtained using non-linear method for the adsorption of IC onto APAN/Fe_3_O_4_–MPA

**Langmuir model**
Maximum adsorption capacity, *q*_m_ (mg g^−1^) = 152.35
Langmuir equilibrium constant, *K*_L_ (L mg^−1^) = 1.83
Adjusted determination coefficient, *R*_adj_^2^ = 0.9820
Standard deviation, SD (mg g^−1^) = 3.89

**Freundlich model**
Freundlich constant, *K*_F_ (mg g^−1^) (L mg^−1^)^1/*n*^ = 82.4
Heterogeneity factor, 1/*n* = 0.19
Adjusted determination coefficient, *R*_adj_^2^ = 0.9333
Standard deviation, SD (mg g^−1^) = 9.82

**Toth model**
Maximum adsorption capacity, *q*_mT_ (mg g^−1^) = 146.2
Toth model constant, *α*_T_ (L mg^−1^) = 0.82
Model exponent, *t* = 0.93
Adjusted determination coefficient, *R*_adj_^2^ = 0.9769
Standard deviation, SD (mg g^−1^) = 4.31

**Table 3:** Comparison of indigo carmine adsorption capacity using APAN/Fe_3_O_4_–MPA composites nanofibers with other reported adsorbents

Material	pH	Dye concentrations (mg L^−1^)	Adsorption capacity (mg g^−1^)	Equilibrium time (min)	Reference
Charcoal from extracted residue of coffee beans	—	10	30	1200	11
Charcoal from rice bran	7	10	9.7	180	10
Chitin	—	10	5.8	—	38
Chitosan	—	90	71.8	120	38
Activated sewage sludge	—	100	60	190	40
Glutaraldehyde cross-linked chitosan	4	30	1.8	200	55
*N*-Vinyl-2-pyrrolidone/acrylonitrile hydrogels	—	50	2.3	7200	56
Calcium hydroxide	12	0.05	0.95	50	6
Mg/Fe layered double hydroxide nanoparticles	9.5	14	55.5	30	57
Activated carbon	2	20	87.8	120	58
Montmorillonite	3	20	40	120	59
PAN/Fe_3_O_4_–MPA composites nanofibers	5	20	154.5	25	This work

The Freundlich expression is based on adsorption onto a heterogeneous surface. The isotherm parameters were calculated using the non-linear form of Freundlich equation, which is given by the following equation;12where *K*_F_ (mg g^−1^) (L mg^−1^)^1/*n*^ is the Freundlich constant related to the adsorption capacity and 1/*n* is the heterogeneity factor. The obtained values of Freundlich parameters are listed in Table 2. The value of 1/*n* was found to be less than unity indicates favorable adsorption process. The values of *R*_adj_^2^ (0.9333) and SD (9.82) indicated that Freundlich model was not appropriate to describe the adsorption experimental data.

The article "Surface modified composite nanofibers for the removal of indigo carmine dye from polluted water" was retracted in 2025. Reasons: duplicated images; unreliable data; unreliable results or conclusions.

Toth isotherm model is used to describe heterogeneous adsorption systems, which satisfies both low and high-end boundary of the concentration. The non-linear equation of Toth model is given as;^38^13where *q*_mT_ is the Toth maximum adsorption capacity (mg g^−1^), *α*_T_ is the Toth model constant (L mg^−1^) and *t* is the model exponent, which is related to heterogeneity of the surface. The model suggests when *t* = 1, the adsorption occurs on a homogeneous surface, and when *t* < 1, the adsorption occurs on a heterogeneous surface. The values of the isotherm constants with *R*_adj_^2^ and SD are given in Table 2. The relative high value of *R*_adj_^2^ (0.9769) and low SD value (4.31) indicated that the isotherm model may use to describe the adsorption experimental data. Also, the Toth component *t* was close to unity, supporting that the adsorption occurred onto a homogeneous surface.

### Influence of pH

The adsorption of IC onto APAN/Fe_3_O_4_–MPA was investigated by varying the pH of the solution over the range of 2–9. The amount of adsorption for IC as a function of pH is shown in Fig. 7. The results obtained clearly indicate that the adsorption process is pH dependent and the maximum adsorption of IC occurs at pH 2–5. The decrease of IC adsorption in higher pH (pH > 6) may be attributed to the increase of repulsive force between the functional groups (–SH) on the surface of APAN/Fe_3_O_4_–MPA and IC, which exists mainly as anion form at higher pH, and thus reduces the adsorption of IC.^43^ The thiol functional groups on the surface of the nanoparticles (Fe_3_O_4_-MPA) may influenced by the pH changes and as a result the thiol interactions with the IC dye may also affected. In order to fabricate the APAN/Fe_3_O_4_–MPA, the surface of APAN nanofibers contains amide (–CONH) and amine (–NH_2_) was coupled with MPA coated Fe_3_O_4_ nanoparticles containing thiol functional groups (–SH). The thiol functional groups on the surface of Fe_3_O_4_ nanoparticles are the prominent sites due to their higher concentration. In acidic solutions (pH = 5), the functional groups of the composite nanofibers would be positively charged (–SH_2_^+^, –CONH_2_^+^and –NH_3_^+^).

**Fig. 7:** Effect of solution pH on the adsorption of IC onto APAN/Fe_3_O_4_–MPA. Experimental conditions: dye initial concentration = 20 mg L^−1^, adsorbent amount = 10 mg, contact time = 60 min. The relative standard deviations of all measurements were less than 5%.

IC also, regardless the solution pH, dissociates into an anionic hydrocarbon compartment having negatively charged sulfonate groups and sodium ions.^44,45^ Therefore, having the oppositely charged species (positive on the nanofibers and negative in the solution), the adsorption process will take effect through electrostatic attraction. However, the anionic compartment of IC also contains N–H groups which have the ability to form hydrogen bonding with either the amide functional group or unreacted primary amines of the nanofibers, which will also facilitate the adsorption process. In our previous work, the pH for point of zero charge (pH_pzc_) of Fe_3_O_4_–MPA nanoparticles was found to be around 7.4.^21^ Thus, Fe_3_O_4_–MPA nanoparticles have positive charge at pH < pH_pzc_ and negative surface charge at pH > pH_pzc_. In case of desorption of IC from the loaded composite nanofibers at basic pH, the functional groups, whether on the surface of Fe_3_O_4_ nanoparticles or on the surface of APAN nanofibers, will be negatively charged (eqn (14))

14 –SH + OH^−^ → –S^−^ + H_2_O

Hence, the electrostatic attraction that caused the IC dye to be adsorbed onto APAN/Fe_3_O_4_–MPA will change to repulsion electrostatic forces between negatively charged functional groups and the anionic compartment of IC dye. This will bring about the dye molecules to be desorbed from the functional groups. Low adsorption at high pH values can be attributed to the presence of some positively charged functional sites as well as the hydrogen bonding and hydrophobic–hydrophobic intercalation of dye molecule with nanofibers Fig. 7. Schematic representation of the suggested mechanism of the adsorption/desorption of IC is shown in Fig. 8. Furthermore, almost complete recovery of IC from APAN/Fe_3_O_4_–MPA was achieved using NaOH solution at pH = 10 (Fig. 9). Therefore, the main mechanism governing the adsorption and recovery of the IC dye is electrostatic attraction and repulsion.

The article "Surface modified composite nanofibers for the removal of indigo carmine dye from polluted water" was retracted in 2025. Reasons: duplicated images; unreliable data; unreliable results or conclusions.

**Fig. 8:** A schematic representation of the proposed mechanism of the interaction of IC with APAN/Fe_3_O_4_–MPA under the experimental conditions studied; (a) adsorption, (b) desorption. Black particles are representative of Fe_3_O_4_ nanoparticles.

**Fig. 9:** Desorption percentage of IC from the loaded APAN/Fe_3_O_4_–MPA as a function of contact time. Experimental conditions: dye initial concentration = 20 mg L^−1^, adsorbent amount = 10 mg, contact time = 60 min, pH = 5, NaOH concentration = 4 × 10^−3^ mol L^−1^. The relative standard deviations of all measurements were less than 5%.

### Regeneration and reuse

The regeneration of the adsorbent is considered as an important parameter and its reuse is considered an economic necessity factor. Therefore, desorption tests were conducted to regenerate the IC dye from loaded APAN/Fe_3_O_4_–MPA and the experiments indicated that a basic solution should be used for effective desorption of IC. Fig. 9 shows the desorption performance of IC from the loaded APAN/Fe_3_O_4_–MPA using low concentration of NaOH solution (4 mmol L^−1^) at pH ∼ 10. Desorption of the IC from the loaded APAN/Fe_3_O_4_–MPA was very fast in the basic solution and 5 min was sufficient to reach the maximum desorption efficiency of 95%.

Furthermore, the APAN/Fe_3_O_4_–MPA was reused in subsequent adsorption–desorption experiments. In these experiments the adsorption efficiency of IC onto APAN/Fe_3_O_4_–MPA was determined from five consecutive adsorption–desorption cycle. The results obtained (Fig. 10) showed that the adsorption efficiency of IC was almost constant in the first four cycles with a slight decrease in adsorption in the fifth cycle, indicating that the regeneration of the APAN/Fe_3_O_4_–MPA was reasonably effective. However, the slight decrease in adsorption in the fifth regeneration cycle may be due to the presence of residues of IC on the composite nanofibers even after fully washing the nanofibers. The ICP measurements of the adsorption and desorption solutions showed no significant amount of iron (<0.1 mg L^−1^) being released into the solution.

The article "Surface modified composite nanofibers for the removal of indigo carmine dye from polluted water" was retracted in 2025. Reasons: duplicated images; unreliable data; unreliable results or conclusions.

**Fig. 10:** Regeneration cycles of APAN/Fe_3_O_4_–MPA. Experimental conditions: initial dye concentration = 20 mg L^−1^, contact time = 60 min, pH = 5, NaOH concentration = 4 × 10^−3^ mol L^−1^.

### Comparative studies

In comparison to the literature, most of the data reported were on the use of photodegradation method for the removal of indigo carmine from solutions. A variety of materials have been tested such as zirconium phosphates,^46^ autoclaved cellular concrete/Fe_2_O_3_,^47^ coal fly ash and zeolite,^48^ 1,10-phenanthrolinium intercalated benotite,^49^ Mg–Al–CO_3_-calcined layered double hydroxides,^50^ TiO_2_-coated non-woven fibers,^51^ MnO_*x*_/TiO_2_ nanoparticles,^52^ and Mn-supported TiO_2_.^53^ However, the reported experiments were either performed in low concentrations of indigo carmine, high amount of adsorbent, high acidity–alkalinity of the dye solution and meanwhile the adsorption capacity for most of the adsorbent materials were relatively low in comparison to our study (Table 3). In the present work the composites nanofibers are flexible and can be suitable for both batch and continuous mode adsorption process. In addition, by tuning the surface functionality on the nanoparticles attached on the surface of the nanofibers, the system will have the ability of selective removal when it comes to multicomponent effluents. On the other hand, photodegradation process lacks the ability to regenerate the adsorbed dye and has the potential of producing toxic elements from dye decomposition which brings about further eco-toxicological investigation. In this study environmental friendly raw material such as iron oxide nanoparticles were used in which they have been utilized in biomedical applications.^54^

## Conclusions

In this work, surface modified APAN/Fe_3_O_4_–MPA composites nanofiber was prepared by electrospinning followed with chemical cross-linking and evaluated for the removal of indigo carmine from aqueous solutions. The results demonstrated that the prepared composite nanofibers showed high adsorption efficiency compared to some other reported adsorbents. Adsorption isotherms reveal that the adsorption mechanism obeys Langmuir model in which monolayer mechanism can be taken in consideration. The adsorption kinetics results showed that the dye adsorption fitted pseudo first order kinetics. The adsorption equilibrium can be reached within 25 min in which it is shorter than other common adsorbents such as activated carbon, charcoal, and chitosan. The strong adsorption ability of the composite nanofibers may attribute to the accessibility for the dye to the active binding sites. The APAN/Fe_3_O_4_–MPA composites nanofibers can be generated and reused several cycles without any significant loss of the adsorption efficiency of indigo carmine. Therefore, the APAN/Fe_3_O_4_–MPA can be considered as a potential adsorbent for the removal of indigo carmine from contaminated water.

The article "Surface modified composite nanofibers for the removal of indigo carmine dye from polluted water" was retracted in 2025. Reasons: duplicated images; unreliable data; unreliable results or conclusions.

## Conflicts of interest

The authors declare that they have no conflict of interest.

## Supplementary Material
